# MOOC and Flipped Classroom Task-Based English Teaching Model for Colleges and Universities Using Data Mining and Few-Shot Learning Technology

This article has been retracted.

**DOI:** 10.1155/2022/9770747

**Published:** 2022-06-13

**Authors:** Yujuan Gong, Jie Zhou

**Affiliations:** ^1^Jiangxi Police Institute, Nanchang, Jiangxi 330013, China; ^2^East China Jiaotong University, Nanchang, Jiangxi 330013, China

## Abstract

As a revolutionary education model, the flipped classroom teaching model has unique advantages over the traditional education model. How to change the teaching method of flipped classroom into a teaching method suitable for college English courses is a problem. The goal of this research is to investigate how to use data mining and few-shot learning technology to investigate the impact of MOOC and flipped classroom task-based college English teaching modes. This work provides a data mining-based decision tree algorithm and examines the enhanced decision tree method. The experimental results of this study demonstrate that two students in each of the two groups believe that the English teaching mode, which is mostly taught by traditional teachers, is very favorable to a thorough understanding of basic knowledge, accounting for 4% of the total. There are 17 students that believe the new teaching methodology is really beneficial, accounting for 34% of the total. This mode was determined to be effective for in-depth knowledge of the basics by a total of 25 students. It can be seen that the flipped classroom model is more popular with students.

## 1. Introduction

Since human beings entered the information society, with the rapid development of information technology, the amount of data generated by human society has also increased dramatically. However, how to turn complicated data into knowledge that people can easily accept and understand is a difficult problem for data researchers. Faced with the situation of “a large amount of data, but little knowledge,” data mining technology came into being. This discipline, which originated in the field of database and artificial intelligence [1], has formed a system and has begun to play a huge role in practical applications.

At present, most mathematics classroom teaching is still not free from the shackles of traditional educational ideas. It has disadvantages such as dogmatization, unification, static, isolation, and separation from the real life of students. The dominant position of students in classroom teaching has not yet been established, lacking due freedom and choice, and there is still a large market for indoctrination education. In recent years, MOOCs and flipped classrooms have entered people's field of vision, which is a new form of educational resources and educational models, which has aroused strong repercussions in the education community around the world. MOOCs mainly use online platforms to display the main educational content in the form of microcourses. The flipped classroom is an innovative and personalized education model. The flipped classroom teaching mode based on MOOC mainly uses network technology and resources to reverse the educational purpose and educational form, educational subjects, and the role of teachers, which has attracted great attention in the field of education.

The innovations of this paper are as follows: (1) It introduces the relevant theoretical knowledge of data mining technology and MOOC and flipped classroom task-based college English teaching mode. It also uses decision tree algorithm based on data mining technology to analyze how data mining plays a role in MOOC and flipped classroom task-based college English teaching mode. (2) Based on the decision tree algorithm, it carried out experiments and analysis on MOOC and flipped classroom task-based college English teaching mode. Through investigation and analysis, it found that the task-based college English teaching model based on MOOCs and flipped classrooms can stimulate students' more interest in learning and enthusiasm for learning.

## 2. Related Work

The rapid development of information technology has brought people a convenient life that was unimaginable before and also impacted the traditional way of cognition of knowledge and information. Jovanovic found that learning strategies are related to flipped classrooms, and he also found that students tend to change the strategies that they employ and switch to less effective strategies. Although the scholar used clustering to discover the problems that students have in learning, he did not propose corresponding solutions based on the students' problems. Yilmaz found that the flipped classroom (FC) teaching model was associated with student satisfaction and motivation. The purpose of his research was to investigate the impact of students' e-learning readiness on student satisfaction and motivation in the FC teaching model. Research was conducted among 20 undergraduate students. They learn using the FC teaching model. The results show that the more satisfied students are, the more active they will be in preparing for the preclass preview. Although the scholar has specific experimental objects, he did not analyze the experimental data [2]. Baytiyeh tried to find out whether the flipped classroom model works in teaching and whether students can acquire skills in this model. Using a qualitative case study design, he found that this type of teaching enriches students' learning experience and helps them develop the skills they need. The scholar proposed a qualitative case study design, but he does not address an actual case [3]. Mcnally et al. found that although the flipped classroom is widely used, it lacks experience and is not easy to be accepted. He surveyed 5 students under the flipped classroom model and the results showed that students can have positive attitudes towards flipped classroom elements according to them. But the scholar came to the result directly, without explaining the whole process [4]. Kostaris et al. found that the emerging flipped classroom method has been widely used in teaching practice and achieved many good results. His main purpose is to design and implement an action study to study the effect of flipped classroom approach in teaching and learning. The scholar did not introduce what this action research is for [5]. Jin et al. found that body recognition is crucial in a variety of applications, including pursuit, defense, and more. Traditional human recognition methods are usually based on vision, biometrics, etc. They proposed a recognition method based on radar micro-Doppler features. The method uses deep convolutional neural networks (DCNNs) [6–8] and can recognize people in contactless, remote, and unilluminated states. But the scholar did not explain why he chose this method.

## 3. Decision Tree Algorithm before and after Improvement Based on Data Mining

### 3.1. The Process and Tasks of Data Mining

Network courses have steadily become an important teaching method in remote education due to the rapid growth of network technology. Students generate a tremendous amount of data about education and learning while taking online courses. Because the knowledge concealed behind the data cannot be mined, the linkages and laws that exist in the data cannot be uncovered when confronted with such a vast data collection. Teachers are unable to comprehend the impact of students' online learning, and studying diverse information points does not enable students to make judgments for themselves. Teachers are unable to improve the content of online courses or the effect of distant education due to their incapacity to alter targeted assistance and the pedagogical structure of online courses in a short amount of time.

Data mining, also known as knowledge discovery in databases, is a hot research topic in the field of artificial intelligence and databases. The so-called data mining refers to the nontrivial process of revealing implicit, previously unknown, and potentially valuable information from a large amount of data in the database. Data mining technology [9] provides an excellent solution to this problem. Data mining is the extraction of hidden data from practical application data that many people do not know in advance and are incomplete and ambiguous. However, it is also a potentially useful information process. Its application of data mining for online course learning is undoubtedly practical. The unearthed knowledge helps teachers to complete higher-level decision-making, adjust the educational structure of online courses in time, and improve the content and educational effects of online courses. The data mining architecture is shown in Figure 1.

As shown in Figure 1: Data mining is the process of mining interesting patterns and knowledge from large amounts of data. The data source is generally a database, data warehouse, Web, etc., and the obtained data is called a data set. Data mining is not a simple job. It does not mean that, with data, using a certain method and building several models, it can get the desired information. Data mining should be a multistep process. Before its implementation, a detailed plan should be made to determine what needs to be done at each step and how to do it. Only in this way can data mining be carried out in an orderly manner and be successful. Different environments and different projects may have different data mining processes [10].

In general, the data mining process goes through the following steps, as shown in Figure 2.

As shown in Figure 2: Knowledge is discovered for application. Now people are using knowledge of the following two methods. One is to look only at the relationships or results described by the knowledge itself to support decision-making, and the other is to analyze knowledge. The knowledge gained will be integrated into the organizational structure of information systems to guide practice. The data mining process is a cyclic process. It will constantly approach the essence of things and achieve the purpose of optimizing and solving problems. It turns useful data into information, information into action, and action into value.

### 3.2. Decision Tree and Related Algorithm Theory

Decision tree is one of the classic methods of data mining. It clearly and completely shows the decision and classification process in a tree structure. The algorithm is simple and intuitive. Decision tree is a decision analysis method to obtain the probability that the expected value of the net present value is greater than or equal to zero by forming a decision tree based on the known probability of occurrence of various situations, to evaluate the project risk, and to judge its feasibility. It is a graphical method that uses probability analysis intuitively. Since this decision branch is drawn as a graph like the branches of a tree, it is called a decision tree.

The properties of a decision tree are that it has a clear hierarchy and logic. The entire decision-making process is straightforward, intuitive, and simple to comprehend, with a good classification effect. However, because the data mining technique involves so many association rules, it is not ideal for clustering [11, 12] and is instead employed for classification. The decision tree method is well suited to processing nonnumeric data, particularly on a large scale. This article is primarily concerned with the use of information such as enrollment sources and college entrance examination results in college and university enrollment. As a result, it primarily describes the information theory-based decision tree classification technique. The schematic diagram of decision tree generation is shown in Figure 3.

As shown in Figure 3: The related concepts in decision tree correlation information theory are as follows:

Information gain reflects the characteristics of the sample [13], and there is a close relationship between the two and a proportional relationship. In probability theory and information theory, information gain is asymmetric, which is used to measure the difference between two probability distributions *P* and *Q*. Information gain describes the difference between coding with *Q* and coding with *P*. Usually *P* represents the distribution of samples or observations, or it may be a theoretical distribution that is precisely calculated. *Q* represents a theory, model, description, or approximation to *P*. The entropy Info(*D*) of data *D* is as formula (1):

(1) $$\begin{array}{c} \text{Info}\left(D\right)=-\sum_{i=1}^{m}P_{i}\log\left(P_{i}\right), \end{array}$$

*P*_*i*_ is the nonzero probability that any information in *D* is contained in class *C*_*i*_.

Attribute *A* is divided into *D* and contains *n* different attribute values 1. From this, it can be obtained that the attribute *A* is divided into *D* into a branch node with *A*={*a*_1_, *a*_2_,…, *a*_*n*_}, *A*={*d*_1_, *d*_2_,…, *d*_*n*_} is a tuple in *D*, and its value in *A* is *a*_*i*_, so the calculation formula of entropy can be obtained as

(2) $$\begin{array}{c} E\left(A\right)=-\sum_{i=1}^{m}\frac{\left|d_{i}\right|}{D}\times \text{Info}\left(d_{i}\right). \end{array}$$

The information gain is the difference between the amount of information before and after, and the calculation formula is

(3) $$\begin{array}{c} \text{Gain}\left(A\right)=\text{Info}\left(D\right)-E\left(A\right). \end{array}$$

The information gain rate regulates the information gain through the parameter value, and the calculation formula is

(4) $$\begin{array}{c} \text{SplitInfo}\left(D\right)=-\sum_{i=1}^{n}\frac{\left|S_{i}\right|}{S}\times \;\log\left(\frac{\left|d_{i}\right|}{D}\right). \end{array}$$

It divides the *n* partitions corresponding to each subset in attribute *A* into the corresponding *D*. The calculation formula of the gain rate can be obtained as

(5) $$\begin{array}{c} \text{GainRation}\left(A\right)=\frac{\text{Gain}\left(A\right)}{\text{SplitInfo}\left(A\right)}. \end{array}$$

There are many algorithms for generating decision trees in data mining. The following focuses on several typical decision tree generation algorithms.

ID3 algorithm is the most influential and typical in decision tree mining [14]. Decision trees classify data for prediction purposes. The decision tree method first forms a decision tree according to the training set data. If the tree cannot give the correct classification for all objects, it selects some exceptions to add to the training set data and repeats the process until the correct decision set is formed. A decision tree represents the tree structure of a decision set.

It sets *G* to be a collection of training instance samples. It assumes that there are *m* classes in *G*; then the expected information to classify a given sample is

(6) $$\begin{array}{c} \text{Inf}\left(g_{1},g_{2},\ldots ,g_{m}\right)=-\sum_{i=1}^{m}\frac{g_{i}}{g}\log_{2}\frac{g_{i}}{g}. \end{array}$$

The expected information obtained by dividing according to the *B* attribute is called the entropy *E*(*B*) of the *B* attribute, which is defined as

(7) $$\begin{array}{c} E\left(B\right)=\sum_{j=1}^{n}\left[\frac{\left(g_{1j}+g_{2j}+\cdots +g_{mj}\right)}{g}\right]\times \text{Inf}\left(g_{1j,\ldots ,}g_{mj}\right). \end{array}$$

The obtained information gain for this partition on the *B* attribute is defined as

(8) $$\begin{array}{c} \text{Gain}\left(B\right)=\text{Inf}\left(g_{1},g_{2},\ldots ,g_{m}\right). \end{array}$$

The ID3 algorithm has the attribute of high information gain, which is the attribute with the highest partition purity in the given attribute set. Therefore, it can calculate the information gain of each attribute of the sample in *G* and obtain the attribute with the maximum information gain as the division attribute [15].

The ID3 algorithm is powerful and easy to use. It seems that this algorithm has been able to cope with most cases of classification applications, but a careful study can find that ID3 is more inclined to generate multibranched attributes when selecting split attributes. In extreme cases, the classification of ID3 algorithm becomes very unreasonable [16]. To this end, some scholars have introduced an extended parameter called segmentation information. It uses this parameter mainly to correct the information gain in the ID3 algorithm. The definition of the extended parameter is as

(9) $$\begin{array}{c} {\text{ExInf}}_{B}\left(G\right)=-\sum_{i=1}^{v}\frac{\left|G_{i}\right|}{\left|G\right|}\log_{2}\frac{\left|G_{i}\right|}{\left|G\right|}. \end{array}$$

It also introduces the gain ratio metric to replace the information gain metric in the ID3 algorithm. It is defined as

(10) $$\begin{array}{c} \text{GainRatio}\left(B\right)=\frac{\text{Gain}\left(B\right)}{{\text{ExInf}}_{B}\left(G\right)}. \end{array}$$

It can be seen that the gain rate not only considers the information gain of the training samples in attribute *B*, but also considers the amount of information generated by the *v* branches generated by the *v* attribute values of attribute *B* [17]. So in the above example, due to the existence of extended parameters, its gain rate tends to be reasonable. The improved algorithm uses the highest gain rate as the splitting attribute, which is more scientific and reasonable [18, 19].

### 3.3. C4.5 Algorithm

C4.5 is a classification decision tree algorithm in machine learning [20]. It combines the advantages of the ID3 algorithm and is continuously improved to better realize the construction of decision trees. C4.5 is a family of algorithms used in classification problems in machine learning and data mining. Its goal is supervised learning. The goal of C4.5 is to learn to find a mapping from attribute values to categories, and this mapping can be used to classify new entities with unknown categories.

It gets the minimum value of the continuity property and stores it in MIN. It also stores the maximum value in MAX and divides the breakpoints *A*_*i*_ in [MIN, MAX] in the continuous attribute:

(11) $$\begin{array}{c} A_{i}=\text{MIN}+\frac{\text{MAX}=\text{MIN}}{N}\times i. \end{array}$$

Assuming that each variable in the database has two distinct values *A* and *B*, the uncertainty assessment of the optimal amount of data, i.e., the information entropy is as

(12) $$\begin{array}{c} S=-\sum_{I}\left(p_{i}\times \mathrm{lg}\left(p_{i}\right)\right). \end{array}$$

There are *V* different data values in the attribute *A* in the set *S*, and *A* is used to divide *S* into *v* subsets, and the information gain rate is calculated during the division as

(13) $$\begin{array}{c} \text{Gain}\left(A_{i}\right)=\text{Gain}\left(A\right)\times \sum_{j\in \left[1,v\right]}p_{i}\log_{2}p_{i}. \end{array}$$

In the data mining algorithm, in order to improve the enthusiasm of the students in class and the learning efficiency, the students' learning progress data set is taken as the research object. This can scientifically apply these potential relevant influencing factors to provide key decision-making basis for future college English teaching [21].

The advantages of the decision tree method include a simple and straightforward analysis, high classification accuracy, and high execution efficiency. As a result, the decision tree technique is highly suited for data mining on a wide scale. ID3 chooses the classification standard for the data it collects. The ID3 algorithm can only mine nonlinear data; hence it chooses split attributes based on the number of attribute values. The C4.5 assessment classification criteria are used to determine the rate of information gain. By gradually increasing the information according to the information gain formula, C4.5 effectively eliminates the issues that emerge in ID3.

### 3.4. C4.5 Algorithm Improvement

The C4.5 decision algorithm has better advantages for mining massive data, and the improved algorithm of the classic C4.5 decision algorithm in the decision tree construction will better construct the decision tree. It places some restrictions on the rules and conventions of data: First, it performs classification based on the constructed new attributes, so it is necessary to centrally process and manage the classification attributes in the dataset. Second, it uses the last generated new attribute to classify, so it needs to pay attention to the approximate accurate rule management with high attribute degree.

The core step of the C4.5 decision tree size algorithm is the attribute selection metric calculation. It needs to compare the information gain of each attribute and select the attribute with the largest value to split the tree. Unfortunately, the logarithmic function is used a lot in entropy calculation, and the calculation of the logarithmic function in almost all programming languages requires a lot of computer computing time. Therefore, the computational efficiency of the algorithm is greatly reduced in each attribute selection. Therefore, the key to solving the problem of computing efficiency is how to optimize the entropy value operation and shorten its operation time. To solve this problem, this paper introduces Taylor's mean value theorem and McLaughlin expansion.

Using the Taylor expansion as a substitution to find the limit of the function is the most widely used. At this time, the Taylor formula containing the Peano remainder is generally used. Other equivalent infinitesimals can also be found using Taylor's formula. Taylor's mean value theorem is

(14) $$\begin{array}{c} f\left(n\right)=f\left(n_{0}\right)+f\prime \left(n_{0}\right)\left(n-n_{0}\right)+\cdots +\theta_{t}\left(n\right). \end{array}$$

It assumes that function *f*(*n*) has a derivative value of order *t* + 1 in a narrow interval around *n*_0_, and *θ*_*t*_(*n*) is Tay's remainder.

Maclaurin's expansion: when *n*_0_=0, Tay's mean value theorem can be converted into Maclaurin's formula, which is

(15) $$\begin{array}{c} f\left(n\right)=f\left(n_{0}\right)+f\prime \left(n_{0}\right)+\cdots +\theta_{t}\left(n\right). \end{array}$$

Among them, when *θ*_*t*_(*n*) is negligible, the following approximate expression is obtained, which is

(16) $$\begin{array}{c} f\left(n\right)\approx f\left(n_{0}\right)+f\prime \left(0\right)m+\cdots +f\prime \left(0\right)\frac{m^{t}}{t}!. \end{array}$$

McLaughlin's formula is a special form of Taylor's formula. It can be seen that, for the logarithmic operation in the entropy value, one can use the approximate expression of McFarland's formula instead. Since there is only the logarithmic operation on the base *e* in the java language, the logarithmic operation in the entropy value needs to be transformed as follows, that is,

(17) $$\begin{array}{c} {\text{Log}}_{2}\left(n\right)=\frac{Ln\left(n\right)}{Ln\left(2\right)}, \end{array}$$

*Ln*(2) is a constant and only needs to be calculated once, while *Ln*(*n*) needs to be improved.

Because *Ln*0=*∞*, function *Ln*(*n*) cannot be directly expanded by McFarland's formula, so people set

(18) $$\begin{array}{c} f\left(n\right)=Ln\left(1+n\right). \end{array}$$

Formula (19) is expanded by the approximate expression 18 of McFarland's formula:

(19) $$\begin{array}{c} f\left(n\right)=Ln\left(1+n\right)\approx \frac{n-n^{2}}{2+n^{3}}+\cdots +\frac{{\left(-1\right)}^{t}n^{t+1}}{\left(t+1\right)}. \end{array}$$

Further approximately, the polynomial (−1)^*t*^*n*^*t*+1^/(*t*+1) can be used to replace the *Ln*(*n*) operation, so as to reduce the computational complexity of the entropy value in the C4.5 algorithm.

### 3.5. The Flipped Classroom Teaching Mode Based on MOOC

With the continuous deepening of reform and opening up, the demand for foreign languages, especially international talents proficient in English, from various industries in society continues to increase. Although the proportion of English in various exams is decreasing, the requirement of English proficiency in the actual fierce competition has not decreased. According to the actual situation, China's college English education reform is being implemented.

In this mode, teachers will use screen recording software to create 10-minute video teaching points and upload them to the Internet. Students can watch in their free time and discover their own problems in time. The video contains a simple class review to deepen students' understanding of the knowledge. The unique method of “students study by themselves before class and practice together in class” is contrary to the previous “teacher lectures in class, students practice after class,” so it is called flipped classroom, as shown in Figure 4.

As shown in Figure 4: The biggest difference between the flipped classroom education model and the previous classroom education model is that, in the flipped classroom, students complete knowledge learning outside the classroom, and the classroom becomes an interactive place between teachers and students. The flipped classroom teaching mode means that students watch teachers' video explanations before or outside of class, and they learn independently, and teachers no longer occupy classroom time to teach knowledge. The classroom becomes a place for teacher-student and student-to-student interaction. It includes answering questions and doubts, cooperative exploration, completing studies, etc., so as to achieve better educational effects. With the support of the network, students can use high-quality educational resources to learn knowledge without relying on teachers. The learning mode of the MOOC is shown in Figure 5.

As shown in Figure 5, a MOOC is a newly imported online course learning medium. It integrates a variety of educational resources, learning management systems, and open network resources, but it differs in several respects from previous online courses. MOOC platforms are open to the general public for free learning as well as formal learners in specialized schools and educational institutions. The construction of curricula and the organization of events are both examples of openness. Anyone can take part in a variety of learning and exchange activities, as well as providing educational resources and themes to the MOOC.

Traditional online course video software is frequently recorded with reference to the classroom teaching form, and the length of the video generally increases. Learners in MOOCs do not receive information passively.

### 3.6. Construction Model of Flipped Classroom Based on MOOC

In a typical flipped classroom teaching mode, preclass activities and in-class activities are the main sections, but these two sections are not separated by the flipped classroom teaching mode. Each section contains specific implementation links. These links reasonably connect the preclass activities with the in-class activities to form a complete and smooth teaching mode. The flipped classroom teaching mode based on MOOC is shown in Figure 6.

As shown in Figure 6, MOOC, a large-scale open online course, is the product of “Internet + education.” It is a newly emerging online course development model. In a typical flipped classroom teaching model, the activities before class and the activities during class are the main parts. These two parts are not separated by the flipped classroom teaching mode. The autonomous learning based on the MOOC platform before class is mainly composed of task bar guided learning module, autonomous learning module, and group module. In the classroom, teachers create appropriate instructional situations based on instructional content, and students complete knowledge internalization through coinvestigation and interaction.

## 4. Decision Tree Algorithm and Experiment and Analysis of Flipped Classroom

### 4.1. Experimental Analysis of Improved Decision Tree Algorithm

In order to simplify the operation, this experiment chooses the first method. It uses the C4.5 original algorithm improved by the previously described improvement scheme. The data used in the experiment comes from the information of 50 students in college English teaching, and the total number of sample instances is 50. In this experiment, the original algorithm and the improved algorithm are compared and analyzed for 5 divisions of the sample instance set, namely, 10, 20, 30, 40, and 50 sample instances. The experimental results are shown in Figure 7.

As shown in Figure 7: It can be seen that, with the increase of the number of data sample instances, the execution efficiency of the improved algorithm is higher. At the same time, in the case of large data sample instance sets, the classification accuracy of the improved algorithm has also been improved to a certain extent. The practice of data mining itself is often faced with the mining of large data set instances. Therefore, using this improved C4.5 algorithm can greatly shorten the waiting time of data analysis and improve work efficiency without sacrificing the classification accuracy. The improved C4.5 algorithm overcomes the deficiencies of choosing attributes with many values when using information gain to select attributes and can complete the discretization processing of continuous attributes.

By comparing the decision trees generated by the two algorithms, it can be known that the improved decision tree shortens the attributes far from the root node by the balance coefficient. This increases the importance of teaching information and makes the classification results more accurate and reasonable. Only a partial decision tree is shown here. The final displayed results are shown in Table 1.

The revised C4.5 method is employed in the subsequent decision tree construction since the improved approach is more reasonable and accurate, as shown in Table 1. The average proportion of leaf node samples of the C4.5 algorithm is 6.6%. The average proportion of leaf node samples of the improved C4.5 algorithm is 7.7%. Because the data used to determine the training set is so tiny, the resulting mining model may have certain flaws. It then validates the training set model against the test set to see if it is accurate. This enables the mining model to be refined and revised further. The decision tree analysis function module of the system module analysis will be used to investigate this.

### 4.2. Experiment and Analysis of Traditional Teaching Mode and MOOC-Based Flipped Church Teaching Mode

This paper analyzes the development trend of English learning in recent years, as shown in Figure 8.

As shown in Figure 8: The study of college English is very important for expanding students' international horizons. The traditional education mode of college English education faces the problems of students' participation and educational effects.

The experimental subjects selected in this experiment are students majoring in English in a university, with a total of 50 people. There are 15 boys and 35 girls. It is divided into two groups, one group is conducted in the traditional teaching mode, which is group A, and the other group is conducted in the flipped classroom teaching mode based on MOOC, which is group B. There are 20 people in each group, and the purpose of this experiment is to change the students' learning attitude and improve the learning enthusiasm of the students in the college English classroom by applying the MOOC-based flipped classroom education model in the college English classroom. After a week of teaching, it first analyzes the students in the traditional teaching mode, as shown in Table 2.

As demonstrated in Table 2, the current teaching mode, which is mostly dependent on instructors' instruction, is unable to pique students' interest in learning, and the majority of students believe that this mode will not improve their learning efficiency or autonomy. Second, the students in group B, who are in the flipped classroom teaching style based on MOOC, are analyzed, as shown in Table 3.

As can be seen from Table 3, there are 9 people who like the MOOC-based flipped classroom teaching model very much, accounting for 45%. Generally, there are 8 people who like it, accounting for 40%. There are 2 people who neither like nor dislike, accounting for 10%. This paper investigates and analyzes two groups of students, as shown in Figure 9.

As shown in Figure 9: Through the summary of the results of the student interview survey, it can be known that the students are more accepting of the new teaching model and have higher satisfaction. This model has improved the overall teaching effect. After the teaching experiment, it tested 2 groups. The weekly test scores of the 2 groups are shown in Tables 4 and 5.

As shown in Tables 4 and 5, the students whose weekly scores in group B were higher than 70 points were significantly higher than those in group A. It can be seen that the new teaching mode has a good teaching effect compared with the traditional teaching mode. The learning ability of group B students has been improved. At the same time, it can also indicate that the students in group B have a significant improvement in the application of knowledge compared with the students in group A.

## 5. Conclusion

Information is becoming a more important driver of humanity's progress in the natural and social sciences. Data mining is a technique for extracting information from seemingly unrelated data that is strongly related to people's lives. The fine-tuning teaching mode is a combination of computer-aided education and network platform technology that compensates for some of the deficiencies of the traditional teaching mode's teacher education mode. The importance of English in worldwide communication is growing, as is the importance of English teaching. MOOCs and flipped classroom task-based college English teaching modes have begun to appear as the traditional teaching mode can no longer match the needs of students. The main focus of this study is on the fundamental concepts of data mining technology, as well as the usefulness of MOOCs and flipped classroom task-based college English teaching modes for future local investigation. It offers a decision tree method based on data mining technology and discovers that decision trees are useful for mining and classifying students' information, resulting in improved English instruction. It conducts experiments on students using various teaching methods in the experimental section. The findings reveal that students prefer the task-oriented collegiate English education strategy based on MOOCs and flipped classrooms. This teaching method boosts students' learning initiative and excitement, as well as their English proficiency.

## Figures and Tables

**Figure 1:** Data mining architecture.

**Figure 2:** Steps of data mining.

**Figure 3:** Schematic diagram of decision tree generation.

**Figure 4:** The difference between the flipped classroom education model and the previous classroom education model.

**Figure 5:** The learning model of MOOCs.

**Figure 6:** The flipped classroom teaching mode based on MOOC.

**Figure 7:** Comparison of algorithms before and after improvement. (a) Comparison of the efficiency of the C4.5 algorithm before and after the improvement. (b) Comparison statistics of C4.5 algorithm classification accuracy before and after improvement.

**Figure 8:** The development trend of learning English from 2020 to 2021.

**Figure 9:** Statistical chart of pre- and posttests of the benefits of the two modes to the mastery of basic knowledge. (a) The traditional teaching mode can stimulate interest in learning. (b) Statistical graph of whether the MOOC-based flipped classroom teaching model can stimulate interest in learning.

**Table 1:** Advantages of the improved decision tree.

Model	C4.5 algorithms	Improved C4.5 algorithm
Tree level	5	5
Number of leaf nodes	15	13
Leaf node sample proportion average	(20/15)/20*∗*100% = 6.6%	(18/13)/18*∗*100% = 7.7%

**Table 2:** Popularity of traditional teaching mode.

Object of investigation	Number of people	Percentage (%)	Effective percentage (%)
Like very much	2	10	10
Generally like	3	15	15
Neither like nor hate	5	25	25
Dissatisfied	8	32	32
Dislike very much	2	10	10

**Table 3:** Popularity of traditional teaching mode.

Object of investigation	Number of people	Percentage (%)	Effective percentage (%)
Like very much	9	45	45
Generally like	8	40	40
Neither like nor hate	2	10	10
Dissatisfied	1	5	5
Dislike very much	0	0	0

**Table 4:** Weekly test scores of group A.

Fraction	Number of people	Percentage (%)	Effective percentage (%)
50–60	3	15	15
60–70	9	45	45
70–80	4	20	20
80–90	3	15	15
90–100	1	5	5

**Table 5:** Weekly test scores of group B.

Fraction	Number of people	Percentage (%)	Effective percentage (%)
50–60	0	0	0
60–70	1	5	5
70–80	7	35	35
80–90	7	35	35
90–100	5	25	25

## Data Availability

The data used to support the findings of this study are available from the corresponding author upon request.
